The article "Low back pain in junior Australian Rules football: a cross-sectional survey of elite juniors, non-elite juniors and non-football playing controls" was retracted in 2011. Reasons: lack of ethics approval or compliance; no approval from the institution.

# Low back pain in junior Australian Rules football: a cross-sectional survey of elite juniors, non-elite juniors and non-football playing controls

**DOI:** 10.1186/1471-2474-11-241

**Published:** 2010-10-19

**Authors:** Wayne Hoskins, Henry Pollard, Chris Daff, Andrew Odell, Peter Garbutt, Andrew McHardy, Kate Hardy, George Dragasevic

**Affiliations:** 1 Department of Chiropractic, Macquarie University, Sydney, NSW 2109, Australia; 2 Harbord Village Chiropractic, Freshwater, NSW 2096, Australia; 3 Norwest Orthopaedic and Sports Physiotherapy, Norwest, NSW 2153, Australia; 4 Enhance Chiropractic and Massage Sports Injury Centre, Ngunnawal, ACT 2913, Australia

## Abstract

**Background:**

Low back pain in junior Australian Rules footballers has not been investigated despite findings that back pain is more prevalent, severe and frequent in senior footballers than non-athletic controls and findings that adolescent back pain is a strong predictor for adult back pain. The aim of this study was to determine the prevalence, intensity, quality and frequency of low back pain in junior Australian Rules footballers and a control group and to compare this data between groups.

**Methods:**

A cross-sectional survey of male non-elite junior (n = 60) and elite junior players (n = 102) was conducted along with a convenience sample of non-footballers (school children) (n = 100). Subjects completed a self-reported questionnaire on low back pain incorporating the Quadruple Visual Analogue Scale and McGill Pain Questionnaire (short form), along with additional questions adapted from an Australian epidemiological study. Linear Mixed Model (Residual Maximum Likelihood) methods were used to compare differences between groups. Log-linear models were used in the analysis of contingency tables.

**Results:**

For current, average and best low back pain levels, elite junior players had higher pain levels (p < 0.001), with no difference noted between non-elite juniors and controls for average and best low back pain. For low back pain at worst, there were significant differences in the mean pain scores. The difference between elite juniors and non-elite juniors (p = 0.040) and between elite juniors and controls (p < 0.001) was significant, but not between non-elite juniors and controls. The chance of suffering low back pain increases from 45% for controls, through 55% for non-elite juniors to 66.7% for elite juniors. The chance that a pain sufferer experiences chronic pain is 16% for controls and 41% for non-elite junior and elite junior players. Elite junior players experienced low back pain more frequently (p = 0.002), with no difference in frequency noted between non-elite juniors and controls. Over 25% of elite junior and non-elite junior players reported that back pain impacted their performance some of the time or greater.

**Conclusions:**

This study demonstrated that when compared with non-elite junior players and non-footballers of a similar age, elite junior players experience back pain more severely and frequently and have higher prevalence and chronicity rates.

## Background

There has been increased awareness of low back pain (LBP) in children and adolescents with several studies showing that LBP is highly prevalent in the early years of life [1,2]. LBP increases with age during the first decades [3], with prevalence increasing significantly following sexual maturity [4]. It has been theorized that LBP in childhood may have important consequences for chronic LBP in adulthood [5]. This theory has been validated with clear correlations between LBP in childhood and adolescence and LBP in adulthood [6]. Hestbaek et al. in a large longitudinal study found LBP in adolescence to be a significant risk factor for LBP in adulthood with odds ratios as high as four [6]. A dose-response association was also demonstrated: the more days with LBP, the higher the risk of future LBP. These findings are supported by research which demonstrates that 90% of schoolchildren with LBP suffer from LBP 25 years later [7].

Questions have been raised regarding LBP at the junior level of sporting competition given that participation in adolescent sports has been found to be a risk factor for LBP [8] and sport participation produces higher LBP prevalence than in non-athletes [9], particularly in males [1]. It is believed that adolescent athletes with less musculoskeletal maturity may be at a heightened risk for more severe and permanent skeletal damage and structural abnormalities, particularly when exposed to years of intense athletic training [10].

There are no specific studies investigating LBP in junior Australian Rules footballers. This is despite the popularity of the sport and recent evidence showing that elite senior and semi-elite footballers experience LBP more severely and frequently than non-athletic controls, with this trend being more evident in elite players [11]. Thus, the primary objective of the present study was to determine the prevalence, intensity, quality and frequency of LBP in junior Australian Rules footballers. The secondary objective was to compare this data between non-elite junior and elite junior participants and with that of a control group of non-footballers.

## Methods

The study was designed as a cross-sectional survey of male junior Australian Rules football participants. Players were drawn from local underage competitions (classified as non-elite junior), the Victorian state based under 18 TAC Cup (classified as elite junior) and a convenience sample of high school students (classified as controls). The study was approved by the Macquarie University Human Ethics Committee.

The Victorian Football League (VFL) was approached by the authors to participate in the study. They agreed and randomly selected 3 TAC Cup teams to provide players for the elite junior group. Non-elite junior players were selected from a convenience sample of junior football clubs from different states. For clubs to consent to participate it was required that they provide access to their entire player rosters to ensure 100% compliance which would assist in providing an accurate reflection of the status of LBP in the participating clubs. The survey was completed during the 2006 season. All players on the playing lists of the selected clubs were invited to participate and complete the survey with responses remaining confidential. Controls were drawn from a convenience sample of male school students, with the specification that they not participate in Australian Rules football.

The study was presented to the clubs and players as a LBP survey. Questionnaires were either administered by an author of the study or by an official representing the participating club, at the preference of the club. In the case of the club wishing to administer the survey, the questionnaires were mailed out along with consent forms and instructions describing the purposes and procedures of the study and how the instruments were to be administered. This was followed by a telephone call to confirm that all procedures would be correctly administered, to ensure players completed every question and to make certain the club officials were qualified to answer questions of the players. None of the assessors were involved in the analysis of the data. Analysis was provided by a person independent to each of the group allocations.

The questionnaire was developed using the validated and reliable Quadruple Visual Analogue Scale (QVAS) [12], the McGill Pain Questionnaire (short-form) (MPQ-SF) [13], along with a series of questions either adapted from an Australian LBP epidemiological study with permission of the author [14] or that the authors developed themselves and thoroughly pilot tested.

The additional questions were:

• How old were you when you had your first ever attack or episode of LBP?

• If applicable, was this a result of your sporting commitments and activities or not related to this?

• When did your current episode of LBP commence?

• If applicable, was this a result of your sporting commitments and activities or not related to this?

• How often do you experience LBP?

• Do you feel that your low back pain negatively effects or impacts your performance?

To assist with answering the questions a diagram of a mannequin that defined the anatomical boundaries of the low back as a shaded area between the last ribs and the gluteal folds was provided. For the purposes of this survey the shaded area represented the low back and subjects were told to focus only on LBP and not other sources of pain. This area was found to be the most commonly used in a review of methodologically sound LBP prevalence studies [15].

The forms were manually entered using Microsoft Excel^® ^and analyzed using GenStat. Descriptive statistics are used to report player characteristics. Linear Mixed Model (Residual Maximum Likelihood) methods were used to compare differences between groups because of imbalance in replication. Log-linear models were used in the analysis of contingency tables. For all tests a p value <0.05 was considered significant, however actual p values are reported in the study.

## Results

Three of the 12 TAC Cup teams, 3 non-elite junior clubs and 2 high schools participated. The subject characteristics of the different groups are shown in table 1. The results of the QVAS questionnaire are presented in table 2. For LBP now, pain levels were significantly different between groups (p < 0.001). For the LBP average and LBP at best, there were significant differences across the three groups (p < 0.001), with no difference between non-elite junior players and controls, but strong differences between them and elite players. For LBP at worst, there were significant differences in the mean pain scores across the three groups (p < 0.001). The difference between elite juniors and non-elite juniors (p = 0.040) and between elite juniors and controls (p < 0.001) was significant, but not between non-elite juniors and controls.

**Table 1:** Descriptive statistics and distribution for the ages of subjects in the study

	Elite junior		Non-elite junior		Control	
Number	102		60		100	

Mean (SD)	17.2 (0.576)		15.8 (0.676)		15.8 (1.237)	

Median	17		16		16	

Range	16-18		14-17		14-18	

	**Frequency**			**Percentage**		

**Age**	**Elite junior**	**Non-elite junior**	**Control**	**Elite junior**	**Non-elite junior**	**Control**

14	0	1	24	0	1.7	24.0

15	0	17	12	0	28.3	12.0

16	10	34	26	9.8	56.7	26.0

17	66	8	35	64.7	13.3	35.0

18	26	0	3	25.5	0	3.0

**Table 2:** Analysis of the Quadruple Visual Analogue Scale (QVAS) questionnaire and results of the overall pain question from the MPQ-SF and frequency of LBP episodes.

QVAS	Elite junior (n = 102)		Non-elite junior (n = 60)		Control (n = 100)	
LBP now mean (SE)	21.32 (2.24)		11.87 (2.02)		6.57 (1.18)	

LBP average mean (SE)	21.68 (1.92)		11.90 (1.60)		11.21 (1.28)	

LBP best mean (SE)	6.50 (1.13)		2.97 (0.94)		1.67 (0.36)	

LBP worst mean (SE)	48.63 (2.83)		39.03 (3.69)		31.71 (2.86)	

	**Frequency**			**Percentage**		

**Overall pain**	**Elite junior** (n = 102)	**Non-elite junior** (n = 60)	**Control** (n = 100)	**Elite junior** (n = 102)	**Non-elite junior** (n = 60)	**Control** (n = 100)

No pain	29	24	41	28.4	40.0	41.0

Mild	43	23	40	42.2	38.3	40.0

Discomforting	24	12	15	23.5	20.0	15.0

Distressing	5	1	4	4.9	1.7	4.0

Horrible	1	0	0	1.0	0	0

**Frequency of pain**	**Elite junior** (n = 102)	**Non-elite junior** (n = 60)	**Control** (n = 100)	**Elite junior** (n = 102)	**Non-elite junior** (n = 60)	**Control** (n = 100)

No pain	8	6	6	7.8	10.0	6.0

Daily	30	7	12	29.4	11.7	12.0

Weekly	9	7	9	8.8	11.7	9.0

Fortnightly	12	8	7	11.8	13.3	7.0

Monthly	11	4	9	10.8	6.7	9.0

3 Monthly	1	4	8	1.0	6.7	8.0

6 monthly	5	5	15	4.9	8.3	15.0

Yearly	26	19	34	25.5	31.7	34.0

The results of the overall pain question are presented in table 2. There were few players with distressing or horrible LBP and the percentage of elite juniors having no pain appeared low.

The results of the MPQ-SF are presented in table 3. Analysing the MPQ-SF, there were no significant differences in the mean sensory values across the three groups (p = 0.068). The difference between elite juniors and non-elite juniors just failed to be significant (p = 0.057). This difference may have been significant had the study had larger subject numbers. There were no significant differences in the mean affective values (p = 0.575) and MPQ-SF total questions (p = 0.112) across the three groups.

**Table 3:** Analysis of the McGill Pain Questionnaire (short form) (MPQ-SF).

MPQ-SF	Elite junior (n = 102)	Non-elite junior (n = 60)	Control (n = 100)	P value between groups
Sensory questions (SE)	14.97 (1.28)	10.95 (1.67)	11.28 (1.29)	0.068

Affective questions (SE)	8.66 (1.38)	6.81 (1.31)	7.05 (1.23)	0.575

Total questions (SE)	13.29 (1.21)	9.84 (1.58)	10.16 (1.22)	0.112

There were a substantial number of players who could not recall when they first experienced LBP (36.3%, n = 37 of elite juniors, 51.7%, n = 31 of non-elite juniors and 41.0%, n = 41 of controls). The mean (SE) age of first onset LBP were: elite juniors 15.18 (0.20), non-elite juniors 13.68 (0.31), and controls 13.88 (0.24). Of the elite juniors, 8.8%, n = 9 said that they had not experienced back pain, 6.7%, n = 4 of non-elite juniors and 18.0%, n = 18 of controls. Using the players who could recall first onset of LBP as being representative of the population, the mean ages of first onset LBP was different across groups (p < 0.001), but there was no difference between non-elite junior players and controls (p = 0.612). The age of first onset LBP for elite juniors was significantly older, by 1.3 years (p < 0.001). When asked whether their first onset LBP was caused by sport or not 71.0%, n = 66 of elite juniors, 66.1%, n = 37 of non-elite juniors and 69.5%, n = 57 of controls indicated that their first onset of LBP was due to sport, although this was non-significant (X^2 ^= 0.39, df = 2, p = 0.821).

With regards to the commencement of the current episode of LBP the probability of a player suffering LBP varied significantly across groups (X^2 ^= 9.71, df = 2, p = 0.008). The chance of suffering LBP increases from 45% for controls), through 55% for non-elite juniors to 66.7% for elite juniors. Defining acute LBP as pain commencing within the last three months, and chronic LBP as pain commencing beyond the last three months then for players who suffer LBP, the probability of LBP being acute is significantly different across groups (X^2 ^= 9.64, df = 2, p = 0.008). The chance that a pain sufferer experiences chronic pain is 16% for controls, and 41% for non-elite juniors and elite juniors. When asked if their current episode of LBP was due to sporting commitments or activities the percentages across groups was not significant (X^2 ^= 5.36, df = 2, p = 0.069). There was no difference in probability that sport was the cause of the current LBP for non-elite juniors and controls (X^2 ^= 0.261, df = 1, p = 0.609) but was significantly more likely for elite juniors (X^2 ^= 5.094, df = 1, p = 0.024).

The frequency of LBP is presented in table 2. The distribution of episodes was different across groups (X^2 ^= 27.27, df = 14, p = 0.018). The difference between non-elite juniors and controls was not significant (X^2 ^= 4.41, df = 7, p = 0.732), while elite juniors were strongly significantly different by comparison (X^2 ^= 22.86, df = 7, P = 0.002).

When the elite junior and non-elite junior players were asked whether LBP impacted their performance there was no statistical significance in distributions (X^2 ^= 3.24, df = 3, p = 0.356). For the elite juniors 33.3%, n = 34 said LBP did not impact their performance, 40.2%, n = 42 said it did little of the time and 21.6%, n = 22 some of the time. For the non-elite junior players 43.3%, n = 26 said LBP did not impact their performance, 26.7%, n = 16 said it did little of the time and 25.0%, n = 15 some of the time.

## Discussion

This study demonstrated that when compared with non-elite junior players and non-football playing school children of a similar age, elite junior Australian Rules football players experience LBP more severely and frequently and have higher prevalence and chronicity rates. Although affected by recall bias and low response rate, the elite junior players experience first time onset LBP at an older age at an age typical of entry into underage elite training programs. The elite juniors did not attribute first time LBP to be due to sporting commitments or activities more so than non-elite junior players or school children. However, sporting commitments or activities were attributed to cause a high percentage of first time LBP in all groups. Elite juniors did attribute sporting commitments or activities to be more likely to cause their current LBP episode. Although there was no difference between the elite junior and non-elite junior players in their belief of whether LBP impacted their performance, both groups had over 25% report that LBP affected their performance some of the time or greater. Of interest, the elite juniors have a prevalence and overall LBP rating the same as semi-elite senior Australian football code participants, using the same research methodology [11].

Strengths of our study include the use of validated questionnaires to quantify the intensity (QVAS) and quality of LBP (MPQ-SF). Functional disability associated with LBP was not determined. This important aspect was not investigated as it was felt that validated questionnaires in use to determine these parameters are not created for elite athletic populations. As far as we are aware, this is the first study to investigate LBP in junior Australian Rules footballers.

Limitations exist in the study conducted. Firstly, the convenience sample taken for the non-football playing school children and non-elite junior players is not a random population sample and may not be representative. However, random sampling not producing a 100% response rate has been discussed as potentially leading to overestimates of LBP in similar research [11,16]. Our controls were used because of their likely non-elite junior sporting participation and likelihood to be matched for age. It should be noted that at school age most children participate in some form of recreational or organised sport either at school or externally. That is why they were termed non-footballers, with the important finding of our study being that their LBP profile largely does not differ from junior footballers. Future study would benefit from documenting what sporting participation, if any, is performed by the control group. Secondly, there was a difference in numbers between the groups, with a larger number of non-elite junior players being preferred. Future study would also benefit from larger total numbers. Thirdly, although ages were close, it was difficult to achieve a complete match between groups, largely due to junior football clubs often finishing before the under 18 level and school children finishing their eduction at an earlier mean age than the elite juniors. Fourthly, as some questions asked were retrospective in nature, there is likely an element of recall bias in the answers to some questions. This is in particular for questions regarding first time onset of LBP, with questions regarding the current episode of LBP being less affected. Lastly, there may be issues with reliability with adolescents competing the questionnaires, although this would have been affected equally between groups.

The older age of onset in LBP of elite juniors is interesting given the increased prevalence, severity, frequency and chronicity in their LBP. A large cross sectional survey has found that adolescents are at a greater risk of LBP if they have low isometric muscle endurance in the back extensors, with no associations found for aerobic fitness, functional strength, flexibility, or physical activity level after adjustment for muscle endurance [17]. It may be that elite juniors are initially protected from LBP due to their increased physical fitness, but this is lost following the excessive spinal loading [9] and high training duration [18] these players face when they enter the elite junior pathway. To support this, sporting participation in the general population is known to result in less frequent LBP, although once LBP is established, sporting participation contributes to increased severity of pain [19]. Elite juniors also face pressure to play and train with LBP (and other injuries) given injuries can affect future selection to professional senior clubs in the Australian Football League (AFL). However, future research would benefit from the inclusion of training and competition volume to more clearly identify its role in the increased incidence of LBP occurring in elite junior footballers. Other potential reasons for the increased incidence of LBP in elite adolescent Australian Rules footballers includes the likely increased prevalence of weight lifting training and the effects that increased loading and training volume may have on the developing skeleton [10].

It has previously been documented that LBP is rarely a self-limiting disorder but characterized by unpredictable variations in pain status, with temporary, rather than permanent remissions [20]. Although these studies are based on adult populations, given that the natural history of LBP in adolescence involves a significantly increased risk of adult LBP, it has been suggested that it might be counterproductive to postpone treatment/prevention until the problems become more severe and chronic [6]. This would require a greater understanding of the knowledge of risk factors for LBP in elite junior Australian Rules footballers along with research investigating prevention and treatment interventions. Hestbaek et al. have suggested a change in focus from the adult to the young population in relation to research, prevention, and treatment of LBP [6]. However, it remains to be seen whether a greater focus on prevention and treatment can eliminate the risk and consequences of future LBP episodes and minimise future chronicity. Future study should assess the potential that LBP has for later career and end of career injury occurring in elite junior players.

Although most LBP is non-specific in nature [1], adolescent athletes presenting with LBP may have a pathologic cause for their symptoms [21]. For this reason, it is important for those caring for younger athletes to maintain a high index of suspicion for some of the more common pathologic causes of LBP in this population. Sports-related diagnoses that must be considered include disc-related back pain, atypical Scheuermann's kyphosis, spondylolysis, and spondylolisthesis [22]. It is unclear whether football code players have a greater prevalence of radiographic lumbar spine abnormalities, including spondylolysis and spondylolisthesis, as age-matched controls [23]. This casts doubts on the usefulness of routine radiographic screening. Other research has documented that junior athletes with chronic LBP form a population of adolescents who have degenerative disc disease (DDD) identified on MRI [24]. For adolescent athletes with DDD, the relative risk of reporting recurrent LBP up to the age of 23 years is 16 compared with those having no disc degeneration [25]. Furthermore, disc protrusion and Scheuermann-type changes also contribute to the risk of persistently recurrent LBP at a later age [25]. LBP in adolescent athletes is a problem that should not be ignored but instead fully evaluated.

Future study should target elite junior footballers to determine whether LBP renders them more susceptible to developing other injuries given LBP in senior footballers produces a 29% increased risk of other injury [26]. Already evidence exists documenting that LBP produces changes in the neuromuscular control of the lumbopelvis [27] and in athletes it produces altered muscle response patterns required for lumbopelvic stabilization during sudden trunk loading following clinical recovery from LBP [28]. These changes in lumbopelvic stabilisation and neuromuscular control could explain the high rates of injuries such as hamstring injuries and groin injuries, which occur in elite junior players [29]. If LBP is determined to be a risk factor for injuries, it should be assessed whether prevention or effective treatment reduces this risk.

Considering that a high percentage of elite junior players stated that LBP impacted their performance some of the time or greater, this should be further investigated. Evidence exists that college level athletes with a history of low back injury with resolved LBP demonstrate significantly diminished athletic performance in a 20 m shuttle run test compared with a healthy group [30]. This is of immense consideration for the elite juniors who get tested for sprint speed and endurance (through a beep test) at the AFL draft camp, results which can affect future career prospects.

## Conclusions

This study demonstrated that elite junior Australian Rules footballers strongly experience LBP more severely, frequently and with higher prevalence and chronicity than non-elite junior Australian Rules footballers and non-football playing school children, who share a similar pain profile. This suggests that Australian Rules football participation is not a risk for adolescent LBP, but elite junior participation is. Future research is required to investigate the consequences of these findings, to determine whether LBP produces a greater risk of other injuries, leads to later or post-career LBP or impacts player performance. In addition, risk factors for elite junior LBP need to be identified along with best practices for prevention and treatment.

## Competing interests

The authors declare that they have no competing interests.

## Authors' contributions

WH conceived the idea of the study. All authors were involved in recruitment of subjects and data entry. WH and HP contributed to writing an initial draft document. All authors contributed to the re-writing of this paper. All of the authors participated in the editing and revisions of the multiple drafts that existed between the initial and final draft. All authors read and approved the final manuscript.

## Pre-publication history

The pre-publication history for this paper can be accessed here:

http://www.biomedcentral.com/1471-2474/11/241/prepub
